The article "Sulforaphane‐induced metabolomic responses with epigenetic changes in estrogen receptor positive breast cancer cells" was published in 2018. Journal: FEBS Open Bio.

# Sulforaphane‐induced metabolomic responses with epigenetic changes in estrogen receptor positive breast cancer cells

**DOI:** 10.1002/2211-5463.12543

**Published:** 2018-11-14

**Authors:** Shuyuan Cao, Li Wang, Zhan Zhang, Feng Chen, Qian Wu, Lei Li

**Affiliations:** ^1^ Department of Hygienic Analysis and Detection and Ministry of Education Key Lab for Modern Toxicology School of Public Health Nanjing Medical University China; ^2^ Department of Epidemiology and Biostatistics and Ministry of Education Key Lab for Modern Toxicology School of Public Health Nanjing Medical University China

**Keywords:** breast cancer, estrogen, hydroxymethylation, metabolism, methylation, sulforaphane

## Abstract

Estrogen is a risk factor for breast cancer. The isothiocyanate sulforaphane (SFN), found in cruciferous vegetables, has been identified as an effective chemopreventive agent, and may prevent or treat breast cancer by reversing estrogen‐induced metabolic changes. Here, we investigated metabolic changes in estrogen receptor‐positive breast cancer (MCF‐7) cells treated with estradiol (E_2_) and/or SFN to identify key metabolite panels that might provide new insights into the underlying mechanisms of the antitumor effects of SFN. Gas chromatography–mass spectrometry and ultra performance liquid chromatography–mass spectrometry (UPLC‐Orbitrap*‐* MS) were used to obtain the metabolic profiles of MCF‐7 cells. The data were analyzed using Student's *t*‐test and multivariate statistics, including principal component analysis and partial least squares discriminant analysis. Hydroxymethylation was detected by UPLC‐Orbitrap*‐* MS and verified by immunofluorescence assay. We report that significant changes in metabolites induced by E_2_ and SFN were associated with differences in glycolysis and energy metabolism, and also amino acid, purine, and folic acid metabolism. E_2_ may alter methylation and hydroxymethylation status via the folic acid pathway. We also identified biomarkers that may be of use in interpretation of the metabolic pathways evoked by the effects of E_2_ and SFN on breast cancer cells. The identified biomarkers associated with metabolic pathways provide new insight into the chemopreventive mechanisms of SFN.

**Abbreviations**
2‐OHE_1/2_: 2‐hydroxyestrone/estradiol
4‐OCH_3_E_1/2_: 4‐methoxyestrone/estradiol
4‐OHE_1/2_: 4‐hydroxyestrone/estradiol
5hmC: 5‐hydroxymethylcytosine
5mC: methylcytosine
C: cytosine
ChIP: chromatin immunoprecipitation
COMT: catechol‐*O*‐methyltransferase
DNMT1: DNA methyltransferase 1
E_1_: estrone
E_2_: estradiol
ER^+^: estrogen receptor positive
ERα: estrogen receptor α
GC‐MS: gas chromatography–mass spectrometry
GSH: glutathione
GST: glutathione‐*S*‐transferase
HMDB: Human Metabolome Database
NQO1: NAD(P)H: quinone oxidoreductase 1
Nrf2: nuclear factor erythroid 2‐related factor 2
PCA: principal component analysis
PLS‐DA: partial least squares discriminant analysis
SFN: sulforaphane
UPLC: ultra performance liquid chromatography
VIP: variable importance in the projection

Estrogen is one of the risk factors associated with breast cancer 1. Two mechanisms for estrogen carcinogenesis have been presented 2. One is estrogen acting through its α‐receptor (ERα) to drive target cell proliferation. 3. The other involves the formation of oxidative metabolites of estrogens, which can react with DNA leading to DNA damage that is responsible for the initiation, promotion, and progression of breast cancer. Estrogen metabolism involves activating and deactivating pathways. The estrogens estrone (E_1_) and estradiol (E_2_) are metabolized to the catechol estrogens, 2‐hydroxyestrone/estradiol (2‐OHE_1/2_) and 4‐hydroxyestrone/estradiol (4‐OHE_1/2_). The resulting reactive quinone metabolites can then react with DNA to form depurinating adducts. These depurinating adducts generate apurinic sites that may induce mutations to initiate breast carcinogenesis. The transformation and tumorigenesis of E_2_ and 4‐OHE_2_ have been observed in human breast epithelial cells (MCF‐10F) lacking ERα and therefore not affected by the presence of anti‐estrogen regents 4. There are also protective mechanisms that maintain the balance between the activating and deactivating pathways. These are methylation of catechol estrogen, conjugation of E_1/2_ quinones with glutathione (GSH), and reduction of quinones back to catechols. The major pathway of detoxification of catechol estrogen is *O*‐methylation catalyzed by catechol‐*O*‐methyltransferase (COMT) 5.

The article "Sulforaphane‐induced metabolomic responses with epigenetic changes in estrogen receptor positive breast cancer cells" was published in 2018. Journal: FEBS Open Bio.

E_2_ also plays an important role in regulating diverse energy metabolic pathways 6, 7 such as glucose transport, glycolysis, the tricarboxylic acid (TCA) cycle/Krebs cycle, mitochondrial respiratory chain, adenosine nucleotide translocator, and fatty acid β‐oxidation and synthesis. Estrogen can also stimulate carbohydrate and fatty acid metabolism 8. Disturbances in the E_2_ metabolic pathways are likely to cause metabolically related diseases such as heart disease, obesity, and estrogen‐dependent breast cancer, of which progression and unresponsiveness to therapy are interrelated.

Sulforaphane (SFN) is an isothiocyanate found in cruciferous vegetables such as broccoli 9. Plant myrosinase and β‐thioglucosidases in gut microflora can hydrolyze the glucosinolate glucoraphanin in broccoli to produce SFN. Many studies have shown that SFN is an effective chemopreventive agent that has anti‐proliferative, anti‐inflammatory, anti‐angiogenic, anti‐metastatic, and anti‐oxidative effects, as well as induction of differentiation, apoptosis, and cell cycle arrest 10, 11, 12, 13, 14. Moreover, SFN can activate the nuclear factor erythroid 2‐related factor 2 (Nrf2) pathway to modulate phase 2 detoxification enzymes, including NAD(P)H: quinone oxidoreductase 1 (NQO1) and glutathione‐*S*‐transferase (GST), as well as act as an epigenetic modifier to regulate *COMT* expression to influence estrogen metabolism^15^, ^16^, ^17^.

Although the biological effects of SFN have partially been studied previously, metabolic pathway responses to SFN in E_2_‐treated breast cancer cells have not yet been investigated. In the present study, we used ultra performance liquid chromatography–mass spectrometry (UPLC‐Orbitrap*‐*MS) and gas chromatography–mass spectrometry (GC‐MS) to evaluate whether SFN could alter the effects of estrogen on major metabolic pathways that are constitutively active, with particular emphasis on tumorigenicity by epigenetic pathway in estrogen receptor positive (ER^+^) breast cancer.

## Materials and methods

### Materials

dl‐Sulforaphane, 17β‐estradiol, and 4‐methoxyestradiol (4‐OCH_3_E_2_) were purchased from Sigma‐Aldrich (St Louis, MO, USA).

### Cell culture

The ER^+^ human breast cancer cell line MCF‐7 was obtained from the American Type Culture Collection (ATCC, Manassas, VA, USA). MCF‐7 cells were cultured as a monolayer in phenol red‐free Dulbecco's modified Eagle's medium (Mediatech Inc., Manassas, VA, USA) supplemented with 5% dextran–charcoal‐stripped fetal bovine serum (Atlanta Biologicals, Lawrenceville, GA, USA). Cells were treated with E_2_ (1 nm), SFN (10 μm), and a combination of E_2_ and SFN for 48 h. Cells treated with DMSO were used as the control. The maximum concentration of DMSO in the culture medium was 0.1% (v/v).

### Sample preparation for metabolomics

The cell culture media were removed by vacuum suction and the cells washed with 2 mL pre‐warmed PBS. Immediately, 1 mL pre‐cooled extraction solution (methanol: water, 4 : 1, v/v) was added. The cells were detached with a cell‐scraper and transferred to a 2 mL centrifuge tube. The plate was washed with 800 μL of extraction solution that was collected into the same centrifuge tube. The cell suspension was further vortexed, quickly frozen in liquid nitrogen for 1 min, and finally stored at −80 °C until analyses.

### GC‐MS metabolomic analyses

Prior to GC‐MS analyses, the cell suspension samples were thawed at room temperature and centrifuged at 17 000 ***g*** for 5 min at 4 °C. A total of 1.5 mL supernatant was then transferred into sample vials and vacuum concentrated to dry in a Labconco (Kansas City, MO, USA) CentriVap system. The dried samples were then derivatized to increase the volatility of polar metabolites. Eighty microliters of methoxyamine (15 mg·mL^−1^ in pyridine) was added to the vials, vortex‐mixed for 30s, and kept in 37 °C for 1.5 h. A total of 50 μL of bis‐(trimethylsilyl)‐trifluoroacetamide, which contained 1% trimethylchlorosilane, was added, and the vial recapped and then vortex‐mixed for 30s. The derivatization procedure was carried out at 70 °C for 1 h.

The article "Sulforaphane‐induced metabolomic responses with epigenetic changes in estrogen receptor positive breast cancer cells" was published in 2018. Journal: FEBS Open Bio.

The analyses of cell extracts were performed on a TSQ‐8000 triple quadrupole GC‐MS (Thermo Fisher Scientific, Bremen, Germany). Separation was operated by a TM‐5MS capillary column (Thermo Fisher Scientific). Helium was used as the carrier gas at a constant flow rate of 1.0 mL·min^−1^. The injector temperature was set at 220 °C. The column temperature was initially set at 80 °C for 2 min and then programmed to ramp up at 10 °C·min^−1^ to 180 °C, 5 °C·min^−1^ to 240 °C, and 25 °C·min^−1^ to 290 °C, and finally held for 9 min. The temperature of the transfer line was set at 260 °C and the ion source temperature was 250 °C. Electron energy was 70 eV and detection was conducted in full scan mode (mass to charge ratio (*m*/*z*) 70–1000).

### UPLC‐Orbitrap‐MS metabolomic analysis

Analyses of the pretreated cell samples were also performed on a UPLC Ultimate 3000 system (Dionex, Germering, Germany), coupled with an Orbitrap mass spectrometer (Thermo Fisher Scientific) equipped with a heated electrospray source at a resolution of 7 × 10^5^ in both positive and negative modes. The operating system was provided by xcalibur 2.2 software (Thermo Fisher Scientific). The separation was performed on a 1.9 mm Hypersil Gold C18 column (100 mm × 2.1 mm; Thermo Fisher Scientific) maintained at 40 °C. A multistep gradient consisting of 0.1% formic acid in water (A) and 0.1% formic acid in acetonitrile (B) was applied. The flow rate of the gradient was 0.4 mL·min^−1^, which was achieved by linearly increasing the concentration of solvent B from 5% to 95% in 15 min, and then sustained with 95% solvent B for 2 min before being re‐equilibrated in 5% solvent B. The UPLC autosampler temperature was set at 4 °C and the injection volume was 5 μL. The operating parameters of the MS were set up as follows: spray voltage of 3 kV, capillary temperature of 300 °C, and flow of the sheath gas, auxiliary gas, sweep gas, and S‐Lens RF level was 40, 10, 2, and 50 arbitrary units, respectively. In the full scan analyses [70–1050 atomic mass units (amu)], the resolution was set at 7 × 10^5^ with an automatic gain control target of 1 × 10^6^ charges, and a maximum injection time of 120 ms. The mass spectrometer was calibrated every 24 h to ensure mass accuracy.

The article "Sulforaphane‐induced metabolomic responses with epigenetic changes in estrogen receptor positive breast cancer cells" was published in 2018. Journal: FEBS Open Bio.

### Metabolomic data analyses

#### Preprocessing analysis of GC‐MS data

All the GC‐MS profiling raw files were converted to common data file format via xcalibur and subsequently processed with the open‐source xcms package operated in the r language (Version 2.11.1; R Foundation for Statistical Computing, Vienna, Austria). Data pretreatment consisted of baseline correction, filtering, peak alignment, matching, and peak normalized processing. The peaks due to column bleed and *N*‐methyl‐*N*‐trimethylsilyltrifluoroacetamide artifacts were excluded from subsequent data analyses. Integrated peak areas of multiple derivative peaks that belonged to the same compound were summed and considered as a single metabolite. The resultant three‐dimensional data, which consisted of annotated peak indices (retention time–*m*/*z* pairs), sample names (observations), and the intensity of each sample (i.e. peak area) were then obtained and introduced into the simca‐p 13.0 software package (Umetrics, Umea, Sweden) for multivariate statistical analyses.

#### The preprocessing analyses of UPLC‐Orbitrap‐MS data

All the UPLC‐Orbitrap‐MS raw data files were produced using sieve software (Thermo Fisher Scientific) where data pretreatment procedures such as baseline correction, peak deconvolution, and peak realignment were performed. This process produced a table organized in a three‐dimensional matrix, including annotated peak indices (retention time–*m*/*z* pairs), sample names (observations), and intensity of each sample (i.e. peak area) for multivariate statistical analyses.

#### Multivariate statistics

The simca‐p 13.0 software package was used for multivariate statistical analyses. All data were mean‐scaled and imported into the software, and an unsupervised principal component analysis (PCA) was applied in order to primarily visualize the overall trend of metabolite profiles between groups. This model helped to reduce the dimensionality of complex high‐dimensional data into two or three components without losing the majority of the bioinformation. However, because it was an unsupervised analysis, it failed to achieve maximum separation and search for variables that counted most in the discrimination between groups. A supervised analysis, a partial least squares discriminant analysis (PLS‐DA), was then performed to optimize classification and search for variables. The variable importance in the projection (VIP) obtained from the PLS‐DA model was useful for achieving the relative contribution of each variable in the classification, such that variables with VIP > 1.3 were considered statistically significant.

The article "Sulforaphane‐induced metabolomic responses with epigenetic changes in estrogen receptor positive breast cancer cells" was published in 2018. Journal: FEBS Open Bio.

#### Selection of potential biomarkers

In order to search for discriminable variables in the two groups, both multivariate and univariate statistics were used. To avoid false discovery rate, a *q*‐test was further applied after Student's *t* test, and variables with VIP > 1.3 and *P* < 0.05 were considered statistically significant as potential biomarkers.

### Genome‐wide 5‐hydroxymethylcytosine and 5‐methylcytosine detection by UPLC‐Orbitrap‐MS

Genomic DNA were extracted by Qiagen (Hilden, Germany) DNeasy Blood & Tissue kit. Three 897 bp DNA standards, each homogeneous for unmodified cytosine (C), 5‐methylcytosine (5mC), or 5‐hydroxymethylcytosine (5hmC), were purchased (Zymo, Irvine, CA, USA), and used to generate a calibration curve. They were enzymatically hydrolyzed to nucleosides by using DNA Degradase Plus (Zymo) 18. Hydrolysate was added with 175 μL 0.1% formaic acid and analyzed by UPLC‐Orbitrap‐MS. Chromatographic separation was the same with the above. The flow rate of the gradient was 0.3 mL·min^−1^ and the injection volume was 10 μL. A multi‐step gradient consisting of 0.1% formic acid in water and methanol was applied, starting with a 4 min gradient of 5–95% methanol, and then sustained with 95% methanol for 2 min before a 2 min re‐equilibration in 5% methanol. Mass spectrometer and operating parameters were the same as above.

### Global 5hmC detection by immunofluorescence

The MCF‐7 cells were grown on coverslips in 35‐mm dishes. After treatment with SFN, the cells were washed in PBS, permeabilized with 0.5% Triton X‐100 in PBS for 15 min, and then fixed with 4% paraformaldehyde for 10 min. The fixed cells were blocked for 30 min in blocking reagent buffer (Beyotime, Shanghai, China) and incubated with primary antibodies in blocking reagent buffer. The primary antibodies and the dilutions used for immunostaining were anti‐5hmC (Active Motif, Carlsbad, CA, USA, no. 39770) antibodies at 1 : 200. After three 5 min washes in PBS, the cells were incubated with Alexa‐488‐labeled secondary antibody (Servicebio, Wuhan, China, GB25301) diluted 1 : 300 in blocking buffer. The nuclei were stained with bisBenzimide H33342 trihydrochloride. Images were captured using a Zeiss (Jena, Germany) LSM 700B confocal microscope. The integrated optical density (IOD) of the annotated nuclei was measured in Image‐Pro Plus 6.0 (Media Cybermetrics, Inc., Rockville, MD, USA). We selected three fields to calculate the IOD value as the following formula: total optical intensity/number of cells in each field.

### UPLC‐Orbitrap‐MS analyses of estrogen metabolite 4‐OCH_3_E_2_

Extraction of 4‐OCH_3_E_2_ from cell pellets was according to our previous procedures 19. Briefly, the cell suspension samples were thawed at room temperature and centrifuged at 7500 ***g*** for 20 min at 4 °C. A total of 1.5 mL metabolite‐containing supernatant was lyophilized in the Labconco CentriVap system. The dried samples were then derivatized, by addition of 500 μL sodium bicarbonate buffer (pH 11.0; 0.2 m) and 500 μL dansyl chloride solution (2 mg·min^−1^ in acetone) to the vials, vortex‐mixed for 30 s, and maintained at 60 °C for 8 min. After derivatization, the mixture was loaded onto Supelclean™ENVI‐18 cartridges (Agilent Technologies, Santa Clara, CA, USA) that were preconditioned with methanol and water. The eluate was lyophilized and re‐dissolved in mobile phase liquid and subjected to UPLC‐Orbitrap‐MS analysis according to our previous procedures 19.

The article "Sulforaphane‐induced metabolomic responses with epigenetic changes in estrogen receptor positive breast cancer cells" was published in 2018. Journal: FEBS Open Bio.

### COMT promoter methylation analysis

Chromatin immunoprecipitation (ChIP) was performed using the ChIP‐IT Express kit (Active Motif) according to the manufacturer's instructions. A total of 10^7^ cells were fixed with 1% formaldehyde and lysed to release chromatin. Chromatin was then enzymatically sheared to obtain chromatin of approximately 100–500 bp using the Active Motif Enzymatic Shearing Kit. Sheared chromatin was immunoprecipitated with antibodies against 5‐mC (Active Motiv, no. 61479). IgG was used as mock control. DNA released from reverse crosslinking was purified prior to qPCR. Starting chromatin was used as input. The level of DNA bound to selected proteins was quantified by SYBR‐Green qPCR using LightCycler^®^96 (Roche, Basel, Switzerland). The primers for the *COMT* gene were 5′‐GCCCATTCACACACACAGTC‐3′ for forward and 5′‐GTTTCATTCCATGCACGACA‐3′ for reverse. The qPCR parameters were 95 °C for 60 s, followed by 45 repeats of 95 °C for 15 s, and 60 °C for 60 s. The level of bound DNA sequences was calculated using the percentage input method ($2^{-[C_{t}\left(\text{ChIP}\right)-C_{t}\left(\text{Input}\right)]}\times 100$, where *C*_t_ is the cycle threshold value) by calculating the qPCR signal relative to input sample.

### Data analysis

All experimental values are presented as the mean ± SD. Besides the multivariate statistics for metabolomics data analyses, comparison between two groups was analyzed by Student's *t* test using prism version 6.0 (GraphPad Software Inc., San Diego, CA, USA). A *P*‐value <0.05 was considered statistically significant. Besides five replicates for UPLC‐Orbitrap‐MS analysis, all experiments were performed with three independent biological replicates.

## Results and discussion

### Metabolomic profiling of MCF‐7 cells treated with E_2_ and/or SFN

Our metabolic profiling was conducted by GC‐MS and UPLC‐Orbitrap‐MS according to the following described conditions. To determine the difference in metabolic pathways between E_2_‐ and SFN‐treated cells, multivariate statistical analysis such as PCA was performed for dimensional reduction. The quality control samples were used to evaluate the stability and repeatability of the equipment. A total of 1199 and 14 809 features were obtained by GC‐MS and UPLC‐Orbitrap‐MS, respectively.

The article "Sulforaphane‐induced metabolomic responses with epigenetic changes in estrogen receptor positive breast cancer cells" was published in 2018. Journal: FEBS Open Bio.

For GC‐MS pre‐treated datasets, a three‐component PCA model, which contained 54.2% of the total variation, was conducted. A relatively good separation among the groups was achieved according to the score plots shown in Fig. 1A. It preliminarily revealed changed metabolic patterns with the different treatments. For further classification, a more complicated PLS‐DA model was performed and the score plots (*R* ^2^ *Y *= 0.99, *Q* ^2^ = 0.786; Fig. 1B) showed that the treated group clearly deviated from the control group. Similarly, a PCA model covering 79.3% of the total variation was obtained from the UPLC‐Orbitrap‐MS datasets (Fig. 1C). The score plots (*R* ^2^ *Y *= 0.987, *Q* ^2^ = 0.735; Fig. 1D) of the PLS‐DA model showed that the groups were distinguished from each other. Moreover, to avoid over‐fitting, a permutation test was performed to further validate the PLS‐DA model. The validation results showed that both permutated tests were lower than the actual test, which demonstrated that the model was robust and had a relatively good predictive power.

**Figure 1:** (A,B) The score plot from PCA (A) and PLS‐DA (B) model of GC‐MS datasets distinguishing among the control, E_2_, and SFN groups. (C,D) The PCA (C) and PLS‐DA (D) score plots of UPLC‐Orbitrap‐MS datasets for pair‐wise comparisons between the control, E_2_, and SFN groups. t[1], principle feature vector; t[2]: the secondary feature vector.

### Potential biomarker identification

The VIP score estimates the importance of each variable in the projection used in the PLS‐DA model, and is used for key variable selection. The variables with both VIP score larger than 1.3 and *P*‐value less than 0.05 were identified as candidate biomarkers.

According to VIP scores and *P*‐values, the variables that significantly changed after E_2_ exposure were selected. Our lab has established an in‐house library within 493 authentic standards with highly accurate *m*/*z* and retention time that were analyzed under the same conditions. Variables without authentic standards were searched for using online commercial databases, including the Human Metabolome Database (hmdb; version 3.6) and Kyoto Encyclopedia of Genes and Genomes (KEGG), and were putatively identified within the limits of 5 parts per million according to metabolite identification confidence defined by the Metabolomics Standards Initiative. The metabolites that were confidently and putatively identified in the samples are listed in Tables 1 and 2, respectively. The results showed that most of metabolites were involved in purine and amino acid metabolism.

The article "Sulforaphane‐induced metabolomic responses with epigenetic changes in estrogen receptor positive breast cancer cells" was published in 2018. Journal: FEBS Open Bio.

**Table 1:** The list of potential biomarkers characterized from GC‐MS

No.	Metabolite^a^	*t*_R_ (min)	VIP score	E_2_ vs control		SFN vs control		E_2_ + SFN vs control		Corresponding metabolic pathway
				Fold change	*P*‐value	Fold change	*P*‐value	Fold change	*P*‐value	
1	l‐Proline	9.15	1.86	1.28	0.0016	0.90	NS	1.16	NS	Arginine and proline metabolism
2	d‐Gluconic acid	19.46	1.80	2.62	0.0060	3.27	0.0001	2.96	0.0081	Energy metabolism
3	*myo*‐Inositol	20.88	1.78	0.80	0.0085	1.31	0.0201	1.18	NS	Galactose metabolism
4	l‐Alanine	6.36	1.77	1.25	0.0096	0.68	0.0072	0.82	NS	Pyruvate metabolism
5	Ethanolamine	8.69	1.72	0.74	0.0159	1.22	NS	0.98	NS	Phospholipid biosynthesis
6	Ribose‐5‐phosphate	21.26	1.61	1.66	0.0371	0.57	0.0280	1.04	NS	Purine metabolism
7	Phosphoric acid	22.59	1.58	1.93	0.0438	0.63	NS	1.26	0.0272	Purine metabolism
8	l‐Aspartic acid	10.77	1.52	0.77	0.06	0.66	NS	0.63	0.0171	Purine metabolism
9	d‐Lactic acid	5.79	1.51	1.13	0.013	1.02	NS	1.08	NS	Pyruvate metabolism
10	Adenosine	28.26	1.33	1.24	NS	0.30	0.001	0.51	0.0194	Purine metabolism

*t*_R_, retention time; NS, not significant.

a Metabolites identified by comparing with the HMDB.

**Table 2:** The list of potential biomarkers characterized from UPLC‐Orbitrap*‐*MS

No.	Metabolite	*m*/*z* (amu)	*t*_R_ (min)	VIP score	E_2_ vs control		SFN vs control		E_2_ + SFN vs control		Corresponding metabolic pathway
					Fold change	*P*‐value	Fold change	*P*‐value	Fold change	*P*‐value	
1	l‐Proline^a^^,^ b	116.0709	0.52	1.79	2.46	0.014	0.39	0.027	1.23	NS	Arginine and proline metabolism
2	Adenine^a^^,^ b	135.0545	0.88	1.64	0.35	0.0119	0.49	0.0419	0.51	NS	Purine metabolism
3	*cis*‐Aconitic acid^a^^,^ b	174.0155	1.59	1.61	2.87	0.0131	1.72	0.0302	1.68	0.0454	Citric acid cycle
4	Arachidonic acid^a^^,^ b	304.2404	10.13	1.60	0.38	0.0105	0.86	NS	0.42	0.0483	Arachidonic acid metabolism
5	Guanosine^a^^,^ b	283.0911	1.23	1.59	4.17	0.0152	0.90	NS	0.97	NS	Purine metabolism
6	4‐Hydroxy‐l‐glutamic acid^b^	161.0308	5.88	1.57	0.35	0.0191	0.88	NS	0.89	NS	Arginine and proline metabolism
7	Folic acid^a^^,^ b	441.1389	4.91	1.49	0.53	0.0492	0.91	NS	0.96	NS	Folate metabolism
8	l‐Arginine^a^^,^ b	175.1188	0.88	1.49	1.26	0.022	0.80	NS	0.91	NS	Arginine and proline metabolism
9	Xanthosine dihydrate^a^^,^ b	284.0761	3.04	1.46	2.88	0.0036	0.21	0.0489	0.89	NS	Purine metabolism
10	8‐Hydroxy‐deoxyguanosine^a^, ^b^	283.0918	1.86	1.43	3.10	0.0142	0.12	NS	0.51	NS	Purine metabolism
11	l‐Tyrosine^a^^,^ b	181.0731	2.02	1.43	2.04	0.0070	0.58	0.0137	0.72	0.0242	Tyrosine metabolism
12	l‐Histidine^a^^,^ b	156.0767	0.78	1.42	1.51	0.047	1.23	NS	1.34	NS	Histidine metabolism
13	l‐Carnitine^a^^,^ b	161.1050	0.72	1.42	1.73	0.0149	0.75	NS	0.88	NS	Fatty acid metabolism
14	Xanthine^a^^,^ b	152.0333	2.77	1.42	2.55	0.0242	0.41	0.0145	1.16	NS	Purine metabolism
15	d‐Ribose^a^^,^ b	1.920863	1.61	1.41	2.13	0.036	1.24	N.S	1.34	NS	Pentose phosphate pathway
16	Deoxyinosine^a^^,^ b	252.0854	6.78	1.40	0.49	0.0427	0.64	NS	0.61	NS	Purine metabolism
17	l‐Glutamine^a^^,^ b	146.0690	0.94	1.39	1.68	0.0272	0.76	0.0180	1.27	0.0324	Purine metabolism

amu, atomic mass unit; *m*/*z*, mass to charge ratio; NS, not significant; *t*_R_, retention time.

a Metabolites identified by comparing with authentic standards.

b Metabolites identified by comparing with the HMDB.

The article "Sulforaphane‐induced metabolomic responses with epigenetic changes in estrogen receptor positive breast cancer cells" was published in 2018. Journal: FEBS Open Bio.

### SFN restored E_2_ treatment‐induced lactic acid and alanine production

In the present study, the E_2_‐treated MCF‐7 cells showed significantly higher levels of l‐alanine and d‐lactic acid than those of cells in control conditions (Table 1 and Fig. 2). Endogenous pyruvate can be converted to lactic acid and also alanine via glutamine–pyruvate transaminase, which is related to the NADH/NAD^+^ ratio, especially as NADH > NAD^+^ 20. During intense exercise, muscle cells do not obtain enough oxygen, so pyruvate is converted to lactic acid and alanine. Anaerobic glycolysis produces cytosolic NADH, which is transported and oxidized in the mitochondria. However, in tumor cells, due to the Warburg effect and increased oxidative stress, energy and glucose are highly consumed even with adequate oxygenation, and cytosolic NADH oxidation does not keep up with glycolytic rates due to limited transfer of cytosolic NADH into mitochondria 21. This resulted in lactic acid and alanine production, which supports gluconeogenesis and also restores NAD^+^ for glycolytic demands. Although we did not measure the glycolytic activity directly, alanine can serve as a good indicator of the rate of glycolysis 22. O'Donnell *et al*. 20 found that the lactic acid/alanine ratio can be used as an index of cytosolic redox status. The ratio of lactic acid to alanine was no different between the control and E_2_‐treated groups (control lactic acid/alanine = 1.61, E_2_‐treated group lactic acid/alanine = 1.47). But the appearance of a slightly higher level of alanine in E_2_‐treated cells may be associated with a reduced cytosolic redox status (low ratio NADH/NAD^+^) or high oxidative status. Accumulated evidence demonstrates that estrogen and estrogen metabolites generate reactive oxygen species, which subsequently generate oxidative stress and enhance phosphorylation of kinases to activate redox‐sensitive transcription factors 23, 24, 25. On the contrary, SFN treatment could restore alanine and lactic acid levels. This suggests that SFN redirected glucose into the Krebs cycle for more efficient metabolism. Additionally, SFN is a natural compound with anti‐oxidant activities, which could activate Kelch‐like erythroid‐derived protein with cap‐n‐collar (CNC) homology‐associated protein 1 (Keap1) and the Nrf2 signaling pathway 15. Moreover, Zhang *et al*. 26 demonstrated that SFN could enhance aerobic glucose oxidation‐related gene expression in mature white adipocytes.

The article "Sulforaphane‐induced metabolomic responses with epigenetic changes in estrogen receptor positive breast cancer cells" was published in 2018. Journal: FEBS Open Bio.

**Figure 2:** The metabolic pathways in response to treatment with E_2_ and/or SFN. The changed metabolites are labelled for up‐regulation, down‐regulation, and unchanged. PRPP, 5‐phosphoribosyl 1‐pyrophosphate.

### E_2_ enhanced purine metabolism and amino acid level to promote tumor growth

The levels of ribose 5‐phosphate, which is involved in the biosynthesis of nucleotides (purines and pyrimidines), and l‐glutamine were increased in the E_2_‐treated group vs the control. Purine metabolites such as adenosine, guanosine, xanthine and xanthosine dihydrate were also increased in MCF‐7 cells treated with E_2_ (Fig. 2). Tumor cellular conditions favoring purines have been shown to enhance the metabolic flux of the *de novo* purine biosynthetic pathway. It was indicated that E_2_ could enhance purine metabolism to promote biogenesis of DNA. Also E_2_ treatment increased the level of amino acids such as l‐proline and l‐arginine in MCF‐7 cells. Purine metabolites and amino acids provide cells with the necessary energy and cofactors to promote cell survival and proliferation and consequently result in tumor progression. In this study, SFN decreased the related purine metabolite and amino acid levels in MCF‐7 cells compared with those in the control. Studies have reported that SFN may regulate cyclin expression to modulate cell cycle control, further to inhibit cell proliferation 17. Our results provided a novel insight into the mechanism by which SFN may regulate purine metabolism and amino acid levels as a cancer chemopreventive agent.

### E_2_ influences methylation status by consuming folic acid

E_2_ treatment can increase global DNA methylation in a process that requires folic acid consumption. Compared to the SFN‐treated group, the level of folic acid in the E_2_‐treated group was very low, which indicated that more folic acid may be consumed with increasing global DNA methylation (Fig. 2). So we measured the global methylation status in MCF‐7 cells treated with E_2_ and/or SFN. Firstly, using UPLC‐Orbitrap‐MS, we determined the global level of genomic 5mC and 5hmC levels in MCF‐7 cells treated with E_2_ and/or SFN. DNA was prepared and digested into the nucleoside components (deoxyribose + base). The mass transitions were monitored at *m*/*z* 258.1079 (5hmC), 242.1129 (5mC), and 228.0972 (C), respectively. UPLC‐Orbitrap‐MS chromatograms of 897 bp DNA standards showed peaks and retention time corresponding to C, 5mC, and 5hmC (Fig. 3). The percentage of 5mC and 5hmC in each sample was expressed as 5mC/C + 5mC and 5hmC/C + 5hmC, respectively. The actual percentage of either 5mC or 5hmC in the amount of deoxycytosine in the samples was 1–5% for 5mC and 0.06–2% for 5hmC, respectively. A comparison of the 5mC and 5hmC levels in MCF‐7 cells treated with E_2_ and/or SFN showed that estrogen may increase the global DNA methylation level, which leads to the repression of DNA repair genes and also of the *COMT* gene. This result was consistent with a previous study 27. Methylated cytosines can be modified to hydroxymethylation (5hmC) by 10,11‐translocation (TET) enzymes 28. 5hmC may act in DNA demethylation to change the methylation status 29. So the methylation change may be based on a metabolomic change and the 5mc to 5hmC transition. Next, 5hmC density was further confirmed by immunofluorescence. Immunostaining of 5hmC was localized in the nuclei of the cells, and was visualized as green‐colored staining (Fig. 4A). As shown, the 5hmC‐specific fluorescence decreased in MCF‐7 cells treated with E_2_, and recovered by SFN treatment. Integrated optical density (IOD) was calculated by image‐pro plus 6.0 software, and green light density in the same number of cells was compared among groups (Fig. 4B). There was a significantly different 5hmC density between the E_2_ and SFN groups. An increase of 5hmC or decrease of 5mC may be associated with genetic instability in SFN‐treated MCF‐7 breast cancer cells, which may regulate the cell cycle. SFN has been already shown to reduce the levels of epigenetic enzymes, such as DNA methyltransferase 1 (DNMT1), in cancer cells 30. Down‐regulated *DNMT1* gene expression could promote the transcription of the *COMT* gene, which accelerates the detoxification of catechol estrogen.

The article "Sulforaphane‐induced metabolomic responses with epigenetic changes in estrogen receptor positive breast cancer cells" was published in 2018. Journal: FEBS Open Bio.

**Figure 3:** (A) UPLC‐Orbitrap‐MS of nucleosides derived from three commercial 897 bp standard DNA fragments showing RT and peaks of C, 5mC, and 5hmC. (B) The ratios of methylated or hydroxymethylated DNA to the total cytosine in the samples. E_2_: 1 nm; SFN: 10 μm. All experimental values are presented as mean ± SD. Comparison between two groups was analyzed by Student's *t* test using prism version 6.0. *P* < 0.05 was considered statistically significant. All experiments were performed with three independent biological replicates.

**Figure 4:** 5hmC‐specific fluorescence in MCF‐7 cells. (A) MCF‐7 cells treated with 1 nm E_2_ and/or 10 μm SFN were immunostained by 5hmC‐specific fluorescent antibody. Nuclei are stained blue, and 5hmC antibody is shown green. (B) IOD value of 5hmC density among groups. The immunofluorescence density of 5hmC is presented as the IOD, the accumulated immunofluorescence density. E_2_: 1 nm; SFN: 10 μm. *P <* *0.05. Scale bar: 20 μm. All experimental values are presented as mean ± SD. Comparison between two groups was analyzed by Student's *t* test using prism version 6.0. *P* < 0.05 was considered statistically significant. All experiments were performed with three independent biological replicates.

### SFN promoted E_2_ conversion to 4‐OCH_3_E_2_ by methylation‐induced regulation of *COMT* gene expression

Catechol estrogens are converted to non‐carcinogenic metabolites such as methoxy‐E_1/2_ by COMT, an important enzyme involved in *O*‐methylation and detoxification of catechol estrogen (Fig. 5). 4‐OHE_1/2_ and quinone metabolites are mutagenic for mammary gland, but 4‐OCH_3_E_1/2_ are considered to be protective and have been shown to inhibit tumorigenesis 31. In the present study, we also measured the levels of 4‐OCH_3_E_2_ at 48 h after E_2_ and/or SFN treatment by UPLC‐Orbitrap‐MS. The results showed that the levels of 4‐OCH_3_E_2_ increased with SFN compared to E_2_ treatment (14.52 ± 1.8 vs 10.9 ± 2.1 pmol/10^6^ cells). In our previous study, we detected the expression and methylation status of a specific gene, *COMT*, in E_2_‐ and/or SFN‐treated MCF‐7 cells. It was found that E_2_ treatment could decrease the expression of *COMT*, which could be reversed by SFN (unpublished data). We speculate that E_2_ and SFN influence the expression of *COMT* through methylation mechanisms. We therefore analyzed the methylation status of the *COMT* gene promoter by ChIP–qPCR. It was shown that E_2_ treatment could increase *COMT* promoter methylation in MCF‐7 cells to decrease *COMT*'s expression, and hence reduced COMT‐mediated detoxification. However, SFN could reverse the E_2_‐induced methylation status (Fig. 6). Studies have shown that SFN can mediate epigenetic alteration 32. In breast cancer cells, SFN suppresses *hTERT* (telomerase reverse transcriptase) expression by impacting the epigenetic pathways including DNMT and histone acetylation at the *hTERT* promoter 16. Altogether, our results demonstrated that the ability of SFN to epigenetically modulate *COMT* expression subsequently influences E_2_ metabolism. Besides the *COMT* gene, SFN also led to induction of *GST* and *NQO1* mRNA to influence E_1/2_‐quinones 33.We found that oxidized glutathione (GSSG) in SFN‐treated MCF‐7 cells was 2.17 times higher than that of the control (*P* < 0.009). It is likely that GST catalyzes the E_1/2_‐quinone conjugation with GSH, which is accompanied by conversion of GSH to GSSG.

The article "Sulforaphane‐induced metabolomic responses with epigenetic changes in estrogen receptor positive breast cancer cells" was published in 2018. Journal: FEBS Open Bio.

**Figure 5:** Pathway for COMT‐induced estrogen metabolism. Estrone (E_1_) and estradiol (E_2_) are preferentially metabolized to form 4‐OHE_1_ and 4‐OHE_2_, respectively. COMT detoxifies 4‐OHE_1/2_ to 4‐OCH_3_E_1/2_. If the activity or expression of COMT is low, catechol estrogens are converted to estrogenic quinone metabolites, and then to DNA adducts, which will result in DNA mutation.

**Figure 6:** *COMT* methylation in MCF7 cells in response to 1 nm E_2_ and 10 μm SFN. Level of methylation of the *COMT* promoter was determined by ChIP–qPCR. The data were normalized by input, and then compared with that in the control. All experimental values are presented as mean ± SD. Comparison between two groups was analyzed by Student's *t* test using prism version 6.0. *P* < 0.05 was considered statistically significant. All experiments were performed with three independent biological replicates.

## Conclusion

In this study, metabolic changes in MCF‐7 breast cancer cells treated with E_2_ and/or SFN were explored in order to find the key metabolic pathways that could provide new insight into the underlying chemopreventive mechanisms of SFN. Significantly changed metabolites induced by E_2_ and/or SFN were involved in glycolysis and energy metabolism, amino acid, purine and folate metabolism. E_2_ and SFN also may influence the epigenetic status of MCF‐7 cells by the folate pathway. It is demonstrated that E_2_ could change the metabolomics responsible for breast carcinogenesis, besides through estrogen‐receptor pathway to alter gene expression. SFN is a promising chemopreventive agent, which may interact with many targets in the cells through multiple pathways. The protective effect of SFN can restore estrogen‐induced damage by a metabolomic pathway or a methylation pathway. Our results illustrated multiple mechanisms for estrogen‐induced metabolic disturbance and methylation changes. In addition, GC‐MS‐ and UPLC‐Orbitrap‐MS‐based metabolomic profiling also led to the discovery of biomarkers that enabled a better interpretation of the metabolic pathways evoked by the effects of E_2_ and SFN on breast cancer cells. However, metabolites were only estimated at the end‐points in our study; therefore, our future work should focus on time‐series metabolomic analyses.

The article "Sulforaphane‐induced metabolomic responses with epigenetic changes in estrogen receptor positive breast cancer cells" was published in 2018. Journal: FEBS Open Bio.

## Author contributions

Conceived and designed the experiments: QW and LL. Performed the experiments: SYC and LW. Analyzed the data: QW, SYC, and ZZ. Contributed reagents/materials/analysis tools: FC and LL. Wrote the paper: SYC and QW. All the authors read and approved the final manuscript.

## Conflict of interest

The authors declare no conflict of interest.
